# The Multilevel Study on the Impact of High-Performance Human Resource Practices on Employees’ Voice Behavior: A Moderated Mediation Model

**DOI:** 10.3389/fpsyg.2022.792329

**Published:** 2022-03-30

**Authors:** Yuanyuan Liu, Dongxu Liu, Hui Du, Shuzhen Liu, Xiaoxue Zhou

**Affiliations:** ^1^School of Management and Economics, Beijing Institute of Technology, Beijing, China; ^2^Management College, Beijing Union University, Beijing, China; ^3^National Transportation Development Institute, Beijing Jiaotong University, Beijing, China

**Keywords:** high performance human resource practices, voice behavior, perceived insider status, voice efficacy, multi-level

## Abstract

Based on the social identity theory, the relationship and influencing mechanism between high-performance human resource practices (HPHRPs) and employees’ voice behavior were explored by constructing a moderated mediation model, and the relationship between the field of human resources and the field of organizational behavior was also established. Through 1,178 paired samples of supervisor-employee survey and multilevel linear model analysis technology, it was found that (1) HPHRPs had a positive impact on employees’ voice behavior; (2) perceived insider status played a mediating role between HPHRPs and voice behavior; (3) voice efficacy played a moderating role between perceived insider status and voice behavior; and (4) voice efficacy played a mediating role in the relationship between “HPHRPs-perceived insider status-voice behavior.”

## Introduction

In the current complicated business environment, ideas and information provided by the employees have been considered important ingredients for managers to make better decisions for the success of the organizations (Liang et al., 2012). The employees’ voice behavior, which has been conceptualized as constructive and challenging ideas and exchanges, has attracted more and more attention by managers due to its feasibility to help organizations identify possible ignored issues, promote organizations to make innovations, and adapt to the dynamical and rapidly changing business environment as well (Yin et al., 2018). Nevertheless, since the voice behavior is not always considered positive, it is a challenge to the current status and might lead to risky consequences, such as the failure of interpersonal relationship. Thus, the employees may feel uneasy and hesitant when expressing their inner thoughts and are not always willing to share their suggestions or opinions with the organization (Detert and Edmondson, 2011). The as-described phenomenon should be paid special attention for the reason that concealing one’s suggestions will be harmful to achieve a “win-win” outcome for both sides of the employers and employees.

At present, extensive studies, regarding the situations and psychological factors that promote or hinder employee’s voice behavior, have been conducted because of recognizing the importance of employees’ voice behavior. However, scholars in the field of human resources and employee relations pointed out that importance should be attached to the micro-process in the study of taking voice as an individual’s pro-social and caring behavior (Barry and Wilkinson, 2015). Barry and Wilkinson (2015) believed that employees’ voice in organizational behavior was unlikely to provide opportunities to challenge macro-level management due to the emphasis on individual discretionary power at the micro-level (Barry and Wilkinson, 2015). Regarding this aspect, scholars in the fields of employee relations and human resources have reached a consensus. They believed that macro-level factors need to be considered, such as high-level strategies, organizational goals, and human resource management practices, in order to have a more comprehensive understanding of employees’ voice (Weller et al., 2019). With the emergence of the strategic human resource management paradigm, high-performance human resource practices (HPHRPs) have become a dominant subject in the discipline of human resource management. HPHRPs regarded the conventional human resource practices as an overall “bundle” or system, rather than fragmented modules, which represented the expression of employees’ collective interests (Ramdani et al., 2014). As a consequence, it is highly necessary to establish a connection between the field of human resources and the field of organizational behavior and integrate the macro- and micro-levels to study voice. Such integration may contribute to coming up with relatively novel insights that help us understand how macro factors drive the psychological mechanism and encourage people to make voice (Mowbray et al., 2015).

According to the social identity theory, everyone has a need for identity. The flexible HPHRPs have the ability to make employees feel the care and attention from the organizations, thereby enhancing the level of perceived insider status. For those individuals with identity, they always regard themselves as the “master” of the organizations, provide positive evaluations to their affiliations, and are willing to put forward voices and suggestions for the development of the organizations (Li et al., 2017). In contrast, there is still a certain gap in the transformation of willingness into behavior. In addition, whether the willingness of employees’ perceived insider status can eventually be transformed into practical voice behavior is also related to the level of individual confidence. The voice efficacy reflected the individual’s confidence in completing the voice behavior, and the people with a high sense of voice efficacy are more willing to transform the identity of the organization into practical voice action.

In this article, a new macro-management factor was explored, taking China as the research background. This factor could not only psychologically drive the voice mechanism but also increase the possibility of employees’ voice behaviors. Specifically, a multilevel mediation model, linking the HPHRPs in the field of strategic human resources with the voice behaviors in the field of organizational behavior, was established. Moreover, the “black box” mechanisms of the two aspects were also investigated from the perspective of social identity.

## Literature Review and Research Hypothesis

### High-Performance Human Resource Practices and Employee Voice

Strategic human resource management is a mode of planning human resource deployment and activities, which aims to promote the organizations to achieve the goals. As a result, strategic human resource adopts systematic viewpoints to test the effects of a series of human resource practices. By this method, the view of strategic human resource management research and the view of traditional human resource function could be well-distinguished (Takeuchi et al., 2010). In the research on strategic human resource management, the concept of HPHRPs has evolved to be a core structure, including the degree to which enterprises invest in attracting, selecting, managing, and retaining the best human capital. At present, under the condition of high demand and competition for employees and management talents, more and more attention has been paid to the potential benefits of employing HPHRPs as an approach to maximize the competitive advantages of enterprises. HPHRPs refer to the combination of a series of separate but closely related human resource management practices, including comprehensive recruitment and selection, widely participated training opportunities, and fully motivated salary system. This series of human resource practices collectively form human resources “bundles,” which aims to improve the performance and the competitiveness of the company *via* enhancing employees’ abilities, attitudes, and motivations (Chadwick and Li, 2019).

Voice behavior, as an informal, autonomous, and upward communication of employees’ thoughts, solutions, or concerns about work-related problems, is a proactive work behavior with the aim of improving the current situation (Jia et al., 2020). Employees’ voice behavior is positively correlated with the expected results, such as personal work performance and organizational effectiveness (Frazier and Bowler, 2015).

Social identity theory illustrates that individuals possess a series of open identities, including personal, organizational, and social identities (Tajfel and Turner, 1979). Each identity reflects one’s sense of self-worth and self-esteem, which in turn act as the basis of cognitive, emotional, and motivational processes. When employees realize that they are a member of the organization, they will give positive assessments and are willing to engage in behaviors that are beneficial to the organization (e.g., voice behavior), even if these behaviors are risky and challenging (Hu and Jiang, 2016). Employees’ perception of the care from the organization lies on the related policies, human resource management practices, as well as the treatment they have previously experienced in the organization. HPHRPs could benefit employees by presenting a fair and open competitive environment, providing opportunities to actively participate in decision-making, and helping them perfect their career planning. Supportive human resource management practices could be regarded as an indication that the organization takes care of its employees. These employees who feel the organization’s care emphasize the common interests, collective welfare, and common goals which inspire the employees to generate identification with the organization. Therefore, it may stimulate employees to actively voice in order to give feedback (Zhu and Akhtar, 2017). Based on the abovementioned statements, the following hypothesis was proposed:

Hypothesis 1: There is a significant positive correlation between HPHRPs and employees’ voice behavior.

### Mediating Role of Perceived Insider Status

With the growing concern for the concept of organizational identification in the field of organizational management, the concept of employees’ perceived insider status has been the research focus by researchers and practitioners. Perceived insider status refers to the extent to which employees regard themselves as a member of a specific organization (Stamper and Masterson, 2002; Li et al., 2018). Although employees’ cognition of the employee-organization relationship was involved in many dimensions, perceived insider status focuses on the degree of employees’ perceived ownership of the organization, which makes up a part of personal social identity (Armstrongstassen and Schlosser, 2011). In reality, existing in the organization and perceived insider identity are two completely different concepts, indicating that employees who are traditionally regarded as “outsiders” by other organization members due to their status (e.g., part-time workers and ethnic minorities) may also feel that they are part of organizational communication. On the contrary, individuals who are currently included in the organization (e.g., full-time employees) may not feel that they are the insiders. It can be learned that employees’ perceived insider status could be changed. Research indicated that both the organizational level [e.g., perceiving the organizational supports (Lapalme et al., 2009) and caring ethical atmosphere (Tan and Liu, 2017)] and the group level [e.g., supports from the leader (Liu et al., 2018) and perceived supports from colleagues (Lapalme et al., 2009)] would be conducive to cultivating employees’ cognition of the identity of insiders.

Social identity theory holds the viewpoint that everyone should seek opportunities to evaluate themselves positively in order to form the qualification of individual group membership or social identity. Social identity contains three parts, namely, social classification, social comparison, and active distinction. Social identity is considered as a kind of cognitive tool, by which, people tend to distinguish and classify the subjects in the surrounding environment, thereby better creating and defining their own positions in the society and making more positive comments on the group that they belong to. Supportive HPHRPs from the organizational level would be beneficial to cultivate employees’ perception of the insiders’ status. Those employees are more likely to behave like citizens and contribute to the success of their teams when they feel that they are well-valued in the work environment (Ma et al., 2019). The reason is that they regard themselves as ingredients of the organization, and they will pay additional attention to the issues to be improved and put forward corresponding constructive suggestions (Chen et al., 2017; Liu et al., 2018). Based on the abovementioned statement, the following hypothesis was put forth:

Hypothesis 2: Perceived insider status plays a mediating role between HPHRPs and voice behavior.

### Moderating Effect of Voice Efficacy

Self-efficacy, an important concept in the field of self-cognition, reflects the confidence in one’s ability to achieve the set goals and represents the degree of individual persistence, effort, and willingness (Bandura, 1986; Koc, 2021). Self-efficacy has the characteristic of domain specificity, and it can be divided into general efficacy and self-efficacy for a specific field (e.g., innovation efficacy and voice efficacy) based on the differences of tasks among different domains. Kish-Gephart et al. (2009) came up with the concept of voice efficacy from the perspective of internal motivation when studying why employees remain silent (Kish-Gephart et al., 2009). The voice efficacy originates from self-efficacy, which is the belief of employees on whether their voice behaviors can be successful, especially whether employees firmly believe that their suggestions will be adopted by the supervisors and contributed to the improvement of organizational performance.

Employees with a relatively stronger sense of voice efficacy always possess strong self-confidence in their behaviors and have strong self-control over things, so they are willing to take the initiative to do their work (Tian and Huang, 2014). After perceiving the sense of “master” of insider identity, employees with a relatively strong sense of voice efficacy will be more eager to voice, so as to improve the disadvantages and deficiencies existing in the current status. Moreover, they will not remain silent because of the decline of their opinions or the ridicules from their workmates. The reason is that they are full of confidence in their voice behaviors, believe that their opinions are constructive and beneficial, and are able to well handle complicated interpersonal conflicts. In contrast, employees with a relatively low sense of voice efficacy are not confident in their suggestions, and they are afraid that their suggestions will be useless or bring troubles to the organizations. Even if they feel that they are part of the organization, they hold extremely resistant or hesitant attitudes to voice behaviors. Based on the abovementioned statements, the following hypothesis was put forth:

Hypothesis 3: Voice efficacy plays a moderating role between perceived insider status and voice behavior.

Furthermore, voice behaviors act as a kind of driving force to make organizational performance realize the efficiency of 1 + 1 > 2. Unfortunately, employees tend to hide their personal thoughts in practical work for their own interests (Zhu and Akhtar, 2017). Not only HPHRPs include specific management measures, but they also pay more attention to the personal feelings of the employees and the formation of a good working atmosphere (Muduli, 2015). With the help of HPHRPs, employees could acquire a fair competitive environment, extensive opportunities to participate in decision-making, reasonable promotion channels, and so on. Individuals with a high sense of voice efficacy would like to trust that their voices could bring fair returns to the organization rather than prejudices or punishments. Besides, after perceiving the created friendly atmosphere, they are more willing to regard themselves as an inside member and make contributions to the development and progress of their organizations. Based on the abovementioned statement, the following hypothesis was put forth:

Hypothesis 4: Voice efficacy plays a mediating role in the process of influencing voice behavior through perceived insider status in HPHRPs.

According to the above analysis, a multilevel moderated mediation theoretical model was proposed, i.e., the HPHRPs at the organizational level affect the employees’ voice behavior by influencing the perceived insider status. This demonstrates that the perceived insider status plays a mediating role between HPHRPs and the employees’ voice behavior. In the meanwhile, the sense of voice efficacy plays a moderated role in the second stage and the whole mediating process. The overall research model is shown in Figure 1.

**FIGURE 1:** Schematic of the research model.

## Research Design

### Research Samples

This study investigated the enterprises in Beijing, Shanghai, Wuhan, Guangzhou, and other places, involving enterprises with attributes, such as production, operation, and construction. To avoid the homologous deviation, the supervisor-employee paired method was employed to collect data, and two questionnaires were also designed. Questionnaire 1 was filled by the employees, including the perception of HPHRPs, perceived insider status, and voice efficacy; Questionnaire 2 was filled by the employees’ direct supervisors, in which the employees’ voice behavior was evaluated by the supervisors. The two sets of questionnaires were numbered and recovered at the same time. In this study, a total of 1,500 paired questionnaires were issued to 60 companies, and finally, feedback from 51 companies was received; 1,178 paired questionnaires were recovered, with a recovery rate of 78.53%.

As can be observed from the investigated employee samples, there were 53.74% of men and 46.26% of women. In the aspect of age, those who aged below 25 years accounted for 20.29%, those who aged in the range of 26–30 years accounted for 21.48%, those who aged in the range of 31–35 years accounted for 20.63%, those who aged in the range of 36–40 years accounted for 16.64%, those who aged in the range of 41–45 years accounted for 13.50%, and those who aged more than 46 years accounted for 0.47%. In the aspect of marital status, married couples accounted for 60.02%, unmarried people accounted for 35.82%, and others accounted for 4.16%. As for the educational background, 23.17% of the investigated employees were below undergraduates, 49.66% of them were undergraduates, 25.72% were post-graduates, and 1.44% were above post-graduates. Regarding seniority in working, 15.79% of the surveyed samples had an experience within 3 years, 38.62% had 3–6 years of experience, 34.04% had 6–9 years of experience, and 11.55% had an experience of more than 10 years.

### Research Tools

In this study, the research scale developed by well-known foreign scholars was adopted. After the translation-back translation process of two PhDs in organizational behavior and the calibration by a professor in organizational behavior, the items with unclear semantics and ambiguities were conducted localized modification, so as to ensure that all the items in the scale could be understood by the survey participants. The five-point Likert-type scale was used in this study (one represented completely disagree and five represented fully agree).

#### High Performance Human Resource Practices

The 28-item scale developed by Su (2010) for Chinese management scenario was adopted, including eight aspects in the scale, e.g., strict recruitment and selection, extensive training, and timely information sharing (Su, 2010). In this study, the internal consistency of the scale Cronbach’s α was 0.85, indicating that it possessed good credibility.

#### Perceived Insider Status

The six-item scale developed by Stamper and Masterson (2002) was adopted, and the topics include “I think I am a member of the company” and “I don’t think I belong to the company” (Stamper and Masterson, 2002). In this study, the internal consistency of the scale Cronbach’s α was 0.86, indicating that it had good credibility.

#### Voice Efficacy

The seven-item scale developed by Duan and Wei (2012) was used, and the topics include “I can seize the opportunity to propose suggestions to the managers” and “No matter in what occasion, I can always express my opinions on the issues in the organization” (Duan and Wei, 2012). In this study, the internal consistency of the scale Cronbach’s α was 0.83, indicating that it had good credibility.

#### Voice Behavior

The 11-item scale developed by Duan and Ling (2011) was employed, which included two dimensions, namely, voice considering the overall situation, and self-aggressive voice (Duan and Ling, 2011). In this study, the internal consistency of the scale Cronbach’s α was 0.81, indicating that it had good credibility.

#### Control Variables

To control the impact of demographic variables on this study, gender, age, marital status, educational background, and working seniority were considered control variables.

### Data Aggregation

In this study, the HPHRPs are an organization-level variable measured by individual units, and it is necessary to aggregate the data at the individual level to the team level. Therefore, the intragroup reliability (*r*_*wg*_) and intragroup correlation coefficient (ICC) were employed to check the compatibility of data aggregation. The results indicated that the intragroup consistency *r*_*wg*_ of HPHRPs was 0.91 (>0.70), the intragroup explanatory variance ratio ICC(1) was 0.08 (>0.05), and the average score reliability of group members ICC(2) was 0.73 (>0.70); all the values reached the acceptable range. The results indicated that the organizational level of HPHRPs aggregated from the individual level was appropriate.

## Results

### Descriptive Statistics and Correlation Analysis

The mean, variance, and correlation coefficient of the four main variables were analyzed using SPSS 22.0 software, and the results are shown in Table 1. It can be seen from the table that HPHRPs were significantly correlated with perceived insider status (*r* = 0.22, *p* < 0.01) and voice behavior (*r* = 0.50, *p* < 0.01), and perceived insider status was significantly correlated with voice behavior (*r* = 0.41, *p* < 0.01). The obtained results preliminarily supported our research expectations.

**TABLE 1:** The mean, variance, and correlation coefficient of the variables.

Variables	*M*	SD	1	2	3
1. HPHRPs	3.36	0.24			
2. Perceived insider status	3.46	0.46	0.20**		
3. Voice efficacy	3.64	1.03	0.22**	0.55*	
4. Voice behavior	3.40	0.95	0.26**	0.41**	0.73**

*p < 0.05, **p < 0.01.

### Confirmatory Factor Analysis

To test the discriminant validity among the variables and the fitting degree of the model, Mplus 7.0 software was used to perform confirmatory factor analysis on the four main variables, and the results are listed in Table 2. The results illustrated that the fitting degree of each indicator of the four-factor model was obviously better than that of other models (χ^2^/*df* = 2.68, Tucker Lewis index (TLI) = 0.91, comparative fit index (CFI) = 0.92, root mean square error of approximation (RMSEA) = 0.06, standardized root mean square residual (SRMR) = 0.06), which demonstrated that the four main variables possessed good discriminant validity.

**TABLE 2:** Results of confirmatory factor analysis.

Model	χ*^2^*	df	χ*^2^/df*	TLI	CFI	RMSEA	SRMR
Single factor model (HPHRPs + PIS + VE + VB)	1023.45	132	7.75	0.65	0.61	0.14	0.14
Two-factor model (HPHRPs, PIS + VE + VB)	853.05	131	6.51	0.73	0.77	0.12	0.13
Three-factor model (HPHRPs, PIS, VE + VB)	543.34	130	4.18	0.81	0.83	0.11	0.11
Four-factor model (HPHRPs, PIS, VE, VB)	345.63	129	2.68	0.91	0.92	0.06	0.06

*HPHRPs, High-performance human resource practice; PIS, Perceived insider status; VE, Voice efficacy; VB, Voice behavior; “ + “ means that the factors are merged into one factor.*

### Hypothesis Test

Since a multilevel model was constructed in this study, HPHRPs belong to the organizational level variable, while perceived insider status, voice efficiency, and voice behavior belong to individual-level variables. Therefore, Mplus 7.0 software was employed to test the direct and indirect relationships among the variables using the hierarchical linear modeling technology.

(1) Zero model. Zero models with perceived insider status or voice behavior as the dependent variable were set to test the between-group variance and within-group variance. The results indicated that the within-group variance of perceived insider status was 0.31, the between-group variance was 0.39, and the between-group variance accounted for 55.71% of the total variance (Model M1); the within-group variance of perceived insider status was 0.43, the between-group variance was 0.37, and the between-group variance accounted for 46.25% of the total variance (Model M4). Therefore, a multilevel regression analysis could be conducted.
(2) Main effect. The analysis results of the hierarchical linear model (HLM) are shown in Table 3. It can be seen from Model M6 that after controlling the control variables, such as gender, age, marital status, educational background, and working time, HPHRPs at the organizational level exhibited a significant positive impact on individual-level voice behavior (β = 0.30, *p* < 0.001). Thus, Hypothesis 1 could be supported.
(3) The mediating role of perceived insider status. Baron and Kenny’s three-step method (1986) was used to test the mediating role of perceived insider status between HPHRPs and voice behaviors. In the first step, the main effects of HPHRPs and voice behaviors have been determined. In the second step, it can be seen from Model 3 that HPHRPs had a significant positive impact on the perceived insider status (β = 0.20, *p* < 0.001). In the third step, it can be seen from Model 7 that when HPHRPs and perceived insider status entered the equation simultaneously, the impact of HPHRPs on voice behavior changed from β = 0.30 (*p* < 0.001) to β = 0.21 (*p* < 0.05). As a result, the mediating role of perceived insider status was tenable. Furthermore, it was not appropriate to use the bootstrap CI estimation method with replacement sampling because the presented model was a multilevel model. Therefore, the mediation effect would be tested again by 20,000 times repeating the Monte Carlo simulations and estimating the CI using R language software. The results illustrated that the 95% CI of perceived insider status was (0.04, 0.09), excluding 0. Based on the above results, Hypothesis 2 could be supported.
(4) The moderating effect of voice efficacy. The moderating effect of voice efficacy between perceived insider status and voice behavior was tested by constructing the interaction items of voice efficacy and perceived insider status. It can be seen from Model 8 that the interaction coefficient of perceived insider status and voice efficacy was significant (β = 0.67, *p* < 0.001). To further demonstrate the moderating function, a diagram of the moderating effect is drawn. As shown in Figure 2, when the voice efficiency was high rather than low, the perceived insider status exhibited a positive effect on the voice behavior. Therefore, Hypothesis 3 could be supported.
(5) Mediating effect with moderation. It can be seen from Table 4 that when the perceived insider status was at a low level (less than 1 SD), the 95% CI of the moderating effect of voice efficacy was (0.03, 0.12); when the perceived insider status was at a high level (higher than 1 SD), the 95% CI of moderating effect of voice efficacy was (0.14, 0.35). Similarly, it was found by Monte Carlo simulations that when the perceived insider status was at a high or low level, there were differences in the mediating role of the perceived insider status between HPHRPs and voice behavior [CI (0.06, 0.25), excluding 0]. Based on the above results, it can be seen that the voice efficacy played a significant moderating role between the indirect effects of “HPHRPs-perceived insider status-voice behavior,” so Hypothesis 4 could be supported.

**TABLE 3:** Multilevel analysis results.

Variable	Perceived insider status			Voice behavior				
	M 1	M 2	M 3	M 4	M 5	M 6	M 7	M 8
Intercept term	2.43	2.45	2.21	2.12	2.51	2.36	2.41	2.68
**Level 1**								
Gender			–0.01		0.03	0.01		0.02
Age		0.10*	0.01		0.04	0.05	0.04	0.03
Marital status		−0.17**	−0.08*		–0.02	–0.01	–0.08	–0.01
Educational background		–0.02	–0.04		–0.03	–0.10	–0.13	–0.04
Working time		–0.05	0.04		0.04	0.05	0.05	0.05
perceived insider status							0.29***	–0.27
Voice efficacy								–0.03
Perceived insider status * Voice efficacy								0.67***
**Level 2**								
HPHRPs			0.20***			0.30***	0.21*	
Within group variance (σ^2^)		0.43	0.37	0.43	0.57	0.52	0.34	0.25
Between group variance (τ_00_)		0.10	0.14	0.37	0.14	0.13	0.34	0.39

*p < 0.05, **p < 0.01, ***p < 0.001.

**FIGURE 2:** Moderating effect of voice efficacy.

**TABLE 4:** Moderated mediating Monte Carlo test.

Moderated variable	Moderated effect	Estimate	95% Confidence interval	
			Upper limit	Lower limit
Voice efficacy	Low perceived insider status	0.32	0.03	0.12
	High perceived insider status	0.17	0.14	0.35
	Difference	0.32	0.06	0.25

## Conclusion and Discussion

### Conclusion

The presented research aims to explore the impact of HPHRPs at the organizational level on employees’ voice behavior at the individual level and, in particular, explore the mediating role of perceived insider status and the moderating role of voice efficacy based on social identity theory. Based on the paired questionnaire survey of 1,178 supervisors and employees from 51 companies, the following conclusions could be drawn.

(1) High performance human resource practices had a positive impact on employees’ voice behavior; (2) the perceived insider status acted as a mediating role between HPHRPs and voice behaviors, i.e., HPHRPs promoted the voice behavior by enhancing employees’ perceived insider status; (3) the voice efficacy played a moderating role between the perceived insider status and voice behaviors, namely, the higher the individual’s voice efficacy was, the better the promotion effect of perceived insider status on voice behavior would be; and (4) voice efficacy played a moderating role in the relationship of “HPHRPs-perceived insider status-voice behavior,” i.e., compared with the individuals with low voice efficacy, those with high voice efficacy were more likely to generate perceived insider status under the influence of HPHRPs, so they were more inclined to produce voice behavior.

### Theoretical Significance

The theoretical contributions of the presented work were listed as follows. On the one hand, a macro factor influencing voice behavior was reported. Scholars in the field of organizational behavior have discovered many personal and organizational factors affecting voice behavior, such as personality, emotion, leadership, and atmosphere perception. In response to the recent calls to consider relatively macro-organizational or management factors to understand employees’ voices (Mowbray et al., 2015), HPHRPs, a representative area of strategic human resource practices, were introduced into the research on individual voice behavior, so as to establish a connection between the field of human resources and the field of organizational behavior (Liu et al., 2017).

On the other hand, the mediating mechanism of HPHRPs affecting voice behavior was proposed from the perspective of social identity. Social exchange theory was mostly adopted in the research on HPHRPs and employees’ initiative behaviors (Miao et al., 2013; Hu and Jiang, 2016). Consistent with these reported outcomes, our study also demonstrated the promotion effect of HPHRPs on employees’ voice behavior. In addition, our study indicated that the perceived insider status could mediate the relationship between HPHRPs and voice behavior from the perspective of social identity. In other words, the integrated HPHRPs could indirectly influence the employees’ voice behavior by enhancing the perceived insider status. Therefore, the influence process of human resource practices on employees’ behavior was not only a social exchange but also a process of self-categorization and self-identification. In the meanwhile, the support of self-voice belief was indispensable when employees chose their own voice tasks. As a proactive behavior, the occurrence of voice required a certain internal push force, which came not only from the reciprocal emotional factors but also from self-identity recognition and self-confidence level assessment. This viewpoint has deepened people’s understanding of the internal effect mechanism of organizational macro factors and employees’ behavior.

### Practical Significance

This study is of important practical significance. First, the organizations should be aware that employee-oriented integrated human resource practices could induce positive responses from the employees. Our results demonstrated that HPHRPs could be regarded as a kind of support to employees and possessed the potential to enhance employees’ voice behavior. For employees, expressing opinions on organizational improvement would be beneficial to formulate and implement human resource practices that could promote personal development (e.g., training, counseling, and other professional development plans) and meet their family needs (e.g., family care plans and other procedures for resolving work-life conflicts).

Second, our findings illustrated that perceived insider status played an important role in transmitting the function of organizational human resource practices to promote voice behavior. This evidence suggested that the managers should think highly of the establishment of employees’ personal identity in the organization, which can be operated through a series of employee-oriented HPHRPs. More importantly, the organization should aware that the voice behavior was risky. For those employees who dared to speak frankly and bluntly, the organization should convey to employees a belief that the value of each employee would be valued and each employee was the “master” of the organization. This sense of recognition was enough for them to bear the risk of voice.

Third, to maximize the effectiveness of HPHRPs, individual differences among employees should be taken into consideration. Our results indicated that voice efficacy significantly distinguished the effectiveness of HPHRPs in establishing perceived insider status and further enhancing voice behaviors. When formulating human resource management of the enterprise, the employees’ voice efficacy should be assessed to evaluate the results caused by these practices. This strategy is conducive to helping the organizations adjust management practices to cater to different groups of employees.

### Limitations and Outlook

Although the proposed hypotheses have been supported to some extent, there are still some limitations in this study. On the one hand, it is related to the cross-sectional design in this study. HPHRPs could influence employees’ voice behavior through perceived insider status, but it takes time for this influence to develop. Moreover, other conclusions could not be excluded even if our research results were consistent with the theoretical hypotheses, and the multisource data (e.g., upper and lower binary paired data) were employed to solve the problems caused by the common method variance to a certain extent (Ye et al., 2020). Therefore, the longitudinal design is recommended in the future study, which may better determine the causal basis of the investigated correlations.

On the other hand, the recent studies regarding voice behavior could be classified into two types, namely, promotional voice and inhibitory voice. The current research focused on voice behavior in a single dimension, while Liang et al. (2012) reported that the risk of inhibitory voice was greater (Liang et al., 2012). Would it have a stronger relationship with management support? This issue is worthwhile to clarify, so as to study whether HPHRPs would exert different effects on promotional or inhibitory voices.

## Data Availability Statement

The original contributions presented in the study are included in the article/supplementary material, further inquiries can be directed to the corresponding author.

## Author Contributions

YL and SL contributed to the idea and wrote the full manuscript. DL and HD collected the data and run the data. XZ revised the full manuscript and proposed improvements. All authors contributed to the article and approved the submitted version.

## Conflict of Interest

The authors declare that the research was conducted in the absence of any commercial or financial relationships that could be construed as a potential conflict of interest.

## Publisher’s Note

All claims expressed in this article are solely those of the authors and do not necessarily represent those of their affiliated organizations, or those of the publisher, the editors and the reviewers. Any product that may be evaluated in this article, or claim that may be made by its manufacturer, is not guaranteed or endorsed by the publisher.
